The article "Effect of Combining Traditional Chinese Medicine with Hormonal Therapy on Quality of Life and Tumor Markers of Prostate Cancer Patients" was published in 2021. Journal: Evid Based Complement Alternat Med.

# Effect of Combining Traditional Chinese Medicine with Hormonal Therapy on Quality of Life and Tumor Markers of Prostate Cancer Patients

**DOI:** 10.1155/2021/5061867

**Published:** 2021-10-13

**Authors:** Pengpeng Gai, Na Li, Min Liu

**Affiliations:** ^1^Department of Traditional Chinese Medicine, Zibo Central Hospital, Zibo 255000, Shandong Province, China; ^2^Department of Traditional Chinese Medicine, People's Hospital of Jinan, Jinan 271100, Shandong Province, China; ^3^Department of Urology, Zibo Central Hospital, Zibo 255000, Shandong Province, China

## Abstract

**Objective:**

To explore the effect of combining traditional Chinese medicine (TCM) with hormonal therapy on the quality of life and tumor markers of prostate cancer patients.

**Methods:**

A total of 60 prostate cancer patients treated in Zibo Central Hospital from June 2017 to June 2021 were selected for the retrospective analysis study and divided into the control group and experimental group based on whether applying TCM treatment, with 30 cases each. The patients in the experimental group received the combined treatment of TCM and hormonal therapy, and those in the control group only accepted the hormonal therapy, so as to analyze their clinical efficacy and tumor marker levels after treatment.

**Results:**

The patients' general information were not statistically different (*P* > 0.05); after treatment, the levels and ratios of total prostate-specific antigen (TPSA) and free prostate-specific antigen (FPSA) of patients in both groups were improved, and the experimental group obtained significantly lower TPSA and FPSA levels (*P* < 0.05) and higher TPSA/FPSA ratios (*P* < 0.05); the incidence of androgen-independent prostate cancer was significantly lower in the experimental group than in the control group (8 vs. 16, *P* < 0.05); in addition, the time to develop into the androgen-independent prostate cancer was longer in patients of the experimental group than those of the control group (*P* < 0.05); the treated patients in the experimental group obtained obviously higher Functional Assessment of Cancer Therapy-Prostate (FACT-P) quality of life scores and Karnofsky score (KPS) than those in the control group (*P* < 0.05), and the number of patients with recovered PSA levels was significantly higher in the experimental group than in the control group (*P* < 0.05).

**Conclusion:**

Combining self-made TCM formula with hormonal therapy can effectively improve the levels of prostate tumor markers and postpone the progress of developing from prostate cancer to androgen-independent prostate cancer, which is conducive to promoting the patients' quality of life.

## 1. Introduction

Although the level of medical diagnosis and treatment in China has been increasing in recent years, cancer, with a high incidence and fatality rate, remains an important disease that threatens human health. Prostate cancer is one of the more frequent cancers in men [1, 2]. According to the regional registration statistics, the incidence of prostate cancer in China ranked the sixth of malignant tumors in men and increases with age [3–6]. Currently, hormonal therapy is an important and effective means of prostate cancer treatment because androgens are the source of prostate cancer cell growth, and cutting off the supply of androgens leads to slow cancer cell growth and even death. In general, hormonal therapy is only effective at the beginning, but most patients will gradually develop hormone-independent prostate cancer, adding difficulties to clinical treatment [7–10]. TCM has gradually accumulated a great deal of clinical practice experiences in the field of tumor treatment and achieved certain efficacy results for a long time, and thus, its value and significance in the treatment of prostate cancer has also received increasing attention, but the relevant mechanisms of action are still in the stage of active exploration [11, 12]. Since 2019, the authors have implemented a comprehensive program of self-made TCM formula combined with hormonal therapy for treating prostate cancer patients, which presents better efficacy, convenient and rapid administration, and high clinical acceptance of patients. To further clarify its efficacy and related mechanism of action, a retrospective analysis study was carried out on the patients treated in our hospital, which is summarized and reported as follows.

## 2. Study Plan

### 2.1. Patient Screening and Grouping

According to the screening criteria for patients, 60 prostate cancer patients treated in Zibo Central Hospital from June 2017 to June 2021 were selected for the retrospective analysis study and divided into the control group and the experimental group based on whether adopting TCM treatment, with 30 cases each. The study was approved by the Ethics Committee of Zibo Central Hospital.

### 2.2. Inclusion Criteria

① The patients met the clinical diagnosis criteria for prostate cancer in the Chinese Standard for Diagnosis and Treatment of Common Malignant Tumors [13]; ② the patients were diagnosed after prostate MRI examination and prostate biopsy pathological examination; ③ the patients met the indications of hormonal therapy; ④ the patients were highly compliant and had complete clinical data; and ⑤ the patients and their family members understood the study and signed the informed consent.

### 2.3. Exclusion Criteria

① The patients presented other severe organic diseases or malignant tumors; ② the condition of the patients was extremely severe and uncontrollable; ③ the estimated survival of the patients was less than 6 months; ④ the patients had severe complications; and ⑤ the patients had communication disorders, limb motor disorders, or cognitive dysfunction.

### 2.4. Methods

All patients received the conventional treatment regimen, and on this basis, those in the control group received the hormonal therapy; i.e., those who were diagnosed with metastasis after general check-up according to the pathological score of prostate biopsy and those who presented surgical indications and received surgery were treated with goserelin acetate (specification: 3.6 mg/tube; manufactured: AstraZeneca UK Limited; registration no. H20100314) and bicalutamide (specification: 50 mg; manufactured: AstraZeneca GmbH; registration no. H20100390) [14–16]. In addition to the hormonal therapy, the patients in the experimental group adopted TCM treatment. To ensure the stable quality of Chinese herbs and avoid affecting the efficacy due to decocting, Huarun Sanjiu TCM concentrate granules were selected, which contained 20 g of prepared *Rehmannia* root, 20 g of common yam rhizome, 15 g of Asiatic Cornelian cherry fruit, 20 g of glossy privet fruit, 20 g of malaytea scurfpea fruit, 20 g of plantain seed, 30 g of tuckahoe, 20 g of Mongolian milkvetch root, 15 g of zhuling, 20 g of paniculate bolbostemma, 30 g of hedyotis, 15 g of black nightshade herb, 10 g of manyleaf *Paris* rhizome, and 15 g of zedoary rhizome. The patients orally took one dose daily with boiled water in two split times (in the morning and evening) after meal, and the total administration time of TCM needed to be over 12 months.

### 2.5. Observation Indexes

Before treatment, the patients' general information including their age, Karnofsky scores (KPS), scores of the fourth edition of Functional Assessment of Cancer Therapy-Prostate (FACT-P), duration of disease, the frequency of chemotherapy, prostate volume, Gleason score, TNM stage, and pathological examination results was recorded.

By drawing patients' blood, their levels and ratios of total prostate-specific antigen (TPSA) and free prostate-specific antigen (FPSA) were measured (with the enzyme-linked immunosorbent assay), and the kits were purchased from Shanghai Tellgen Life Science Co., Ltd. (NMPA Certified No. 20153401695/NMPA Certified No. 20153401809); mean time for developing from advanced prostate cancer to androgen-independent prostate cancer and the number of affected patients were recorded.

The quality of life of the prostate cancer patients was evaluated by the FACT-P scale, which included 12 items and mainly evaluated the prognostic quality of life from the dimensions of patients' physical well-being, social/family well-being, emotional well-being, functional well-being, and prostate cancer subscale, with higher scores indicating better quality of life; the patients' performance status was evaluated by the KPS scale, with higher scores indicating that the patients had better physical health and could bear some adverse reactions caused by treatment; see Table 1 for the specific scoring standards. The patients' prostate-specific antigen (PSA) levels were measured, and the clinical observation point was 4 ng/ml; i.e., less than 4 ng/ml was considered as normal, and PSA between 4 and 10 ng/ml was called the gray interval.

### 2.6. Statistical Processing

In this study, the between-group differences in data were calculated by the SPSS22.0 software, the picture drawing software was GraphPad Prism 7 (GraphPad Software, San Diego, USA), the items included were the enumeration data and the measurement data, which were expressed by (n (%)) and ($\bar{\text{x}}$ ± *s*) and examined by the *X*^2^ test and *t*-test, respectively, and differences were considered statistically significant at *P* < 0.05.

## 3. Results

### 3.1. General Information

After statistical processing, no statistical differences in the patients' general information between the two groups were observed (*P* > 0.05). See Table 2 for specific values.

### 3.2. Levels and Ratios of TPSA and FPSA

After treatment, the levels and ratios of TPSA and FPSA in patients of both groups were improved, and the experimental obtained significantly lower TPSA and FPSA levels (*P* < 0.05) and higher TPSA/FPSA ratios (*P* < 0.05) than the control group, indicating statistically significant differences. See Table 3.

### 3.3. Situation of Developing into Androgen-Independent Prostate Cancer

The incidence of androgen-independent prostate cancer was significantly lower in the experimental group than in the control group (8 vs. 16, *P* < 0.05); in addition, the time to develop into the androgen-independent prostate cancer was longer in patients of the experimental group than that in patients of the control group (*P* < 0.05). See Table 4.

### 3.4. FACT-P Quality of Life Scores and KPS Scores

After treatment, the experimental group obtained obviously higher FACT-P quality of life scores and KPS scores than the control group (*P* < 0.05); see Figure 1 for specific data.

### 3.5. PSA Level

After treatment, the number of patients with PSA level restored to normal was significantly higher in the experimental group than in the control group (*P* < 0.05); see Table 5.

## 4. Discussion

Prostate cancer is a cancer specific to men, with cancer cells either growing slowly and leading to late onset or growing rapidly and difficult to control, seriously threatening the physical health and quality of life of a large number of men. Hormonal therapy is the usual means of treating prostate cancer in the clinic, which mainly includes orchiectomy and the use of antiandrogen drugs and GnRH-agonist. Generally, hormonal therapy has better short-term outcomes, but in the longer term, its efficacy mainly rests with the androgen dependence of cancer cells; i.e, the higher the dependence, the better the inhibitory effect on cancer cells of the therapy [17–20]. Based on the analysis on TCM theory, the authors believe that prostate cancer is a renal disease, which is mostly found in middle- and old-aged men, and prostate cancer patients mainly have dysuria, rectal pain, hematuria, and other symptoms accompanied by different degrees of lumbar, hip, and lower abdominal pain, which are associated with dysfunctions of the kidney storing essence, kidney governing water, and kidney governing bones. Medium-elderly male patients mostly suffer from deficiency of kidney essence, blockage of sanjiao and shuidao, disorder of bladder functioning, poor drainage of lower jiao water, and stagnation of fluid-dampness, which, after a long time, will produce phlegmatic toxin that blocks meridian and qi-blood circulation and then generates blood stasis, and finally, intermingled phlegm and stasis will block the seminal orifice and lead to prostate cancer. Therefore, TCM mainly treats prostate cancer by invigorating the kidney and using the Chinese herbs with the efficacy of being antitumor, promoting blood circulation to remove blood stasis, and removing phlegm to promote diuresis because the tumorigenesis is associated with phlegm and stasis. Combined with part of clinical experience, a comprehensive program of self-made TCM formula combined with hormonal therapy for prostate cancer patients was implemented by the authors to make up for the shortage of hormonal therapy and try to balance the treatment of prostate cancer, thereby guiding future prognosis and improving the quality of life for patients.

In this study, the levels and ratios of TPSA and FPSA of patients in both groups were improved after treatment, and the experimental group obtained significantly lower TPSA and FPSA levels (*P* < 0.05) and higher TPSA/FPSA ratios (*P* < 0.05) than the control group; it was found that prostate epithelial cells could secrete a protease, the specific antigen, which was very low in normal body serum but would be significantly elevated in patients with prostate cancer due to the destruction of normal prostate tissue. The results were consistent with the study results of Khachaturov [21], which proved that, on the basis of hormonal therapy, the combined application of self-made TCM formula could effectively inhibit the specific antigen levels in patients with prostate cancer and present significant efficacy. The incidence of androgen-independent prostate cancer was significantly lower in the experimental group than in the control group (8 vs. 16, *P* < 0.05), in addition, the time to develop into the androgen-independent prostate cancer was longer in patients of the experimental group than that in patients of the control group (*P* < 0.05), implying that combining the self-made TCM formula with hormonal therapy presented a certain efficacy in treating prostate cancer, especially in prolonging the transformation to androgen-independent prostate cancer. After treatment, the FACT-P quality of life scores and KPS scores of patients were obviously higher in the experimental group than in the control group (*P* < 0.05), indicating that performing additional TCM treatment could improve the overall physical condition of prostate cancer patients, alleviate the symptom impact, and promote quality of life. The number of patients with PSA level restored to normal after treatment was significantly higher in the experimental group than in the control group (*P* < 0.05). PSA, a serine proteinase involved in sperm and semen formation, is derived from the epithelial cells of the prostatic duct and acinus and often used for the identification of benign and malignant neoplasms and as the important indicator in the postoperative follow-up to determine the progression of the disease and the condition of surgical treatment. This study demonstrated that the effect of combined treatment with TCM on PSA was more obvious.

In the hormonal therapy, bicalutamide is an antiandrogen agent that achieves the purpose of treatment by preventing the action of endogenous androgens on the prostate, and goserelin acetate is a GnRH-agonist that can cause a dramatic increase in testosterone in early treatment, exert a combined effect with bicalutamide, and block androgens after testosterone decrease, thereby inhibiting tumor growth. However, side effects may occur in patients after hormonal therapy, which mostly belong to deficiency of both the kidney and spleen, as well as qi and yin. It is described in Huangdi Neijing that “With vital qi inside, your body will not be affected by pathogenic qi” and “Attack of pathogen will lead to deficiency of qi.” TCM treatment is dominated by supporting healthy energy to eliminate pathogenic factors, which can improve patients' immunity and alleviate the side effects of chemoradiotherapy, while also having an important role in ameliorating cancer symptoms and protecting immune system function, and thus, combining TCM with Western medicine in the treatment of malignant tumors has attracted much attention [22–25]. The TCM formula herein can strengthen kidney and spleen, invigorate qi and yin, and ameliorate the side effects from hormonal therapy, which presents the overall efficacy of strengthening vital qi with the additional effects including clearing heat and removing toxicity, promoting blood circulation to remove blood stasis, diuresis, and diffusing dampness, and dissipating phlegm and resolving masses. In the formula, paniculate bolbostemma, hedyotis, black nightshade herb, manyleaf *Paris* rhizome, and zedoary rhizome are Chinese herbs with the effects of clearing heat, removing toxicity and diuresis, and promoting blood circulation to remove blood stasis and have the direct effects of anti-inflammation and antitumor demonstrated in pharmacological research; in addition, the herbs including malaytea scurfpea fruit, Asiatic Cornelian cherry fruit, glossy privet fruit, and plantain seed can ameliorate patients' symptoms such as dysuria, and pharmacological research demonstrated that they have the estrogen-like effect and act synergistically with hormonal therapy drugs to resist the androgen activity; particularly for those with intractable prostate cancer, they can mildly strengthen the renal yang, greatly nourish the renal qi, relieve the clinical symptoms, and improve the quality of life; using prepared *Rehmannia* root, common yam rhizome, Asiatic Cornelian cherry fruit, glossy privet fruit, malaytea scurfpea fruit, tuckahoe, zhuling, plantain seed, Mongolian milkvetch root, and other herbs together can invigorate the kidney for nourishing semen and strengthen the spleen to invigorate qi, improve the systematic symptoms in patients, and enhance the body immunity; some of the kidney-nourishing herbs also have the functions of bidirectionally regulating the hypothalamic-pituitary-adrenal axis (HPA axis), ameliorating the side effects caused by hormonal therapy and prolonging the time for patients to progress to androgen-independent prostate cancer. This study also has the following deficiencies. For example, the sample size was small due to the limited research cost, so a multicenter study with larger sample size is still in need. In addition, the follow-up period was short, and statistics on the long-term survival of the patients were lacking.

In conclusion, the combination of self-made TCM formula and hormonal therapy effectively improves the prostate tumor marker levels in patients with prostate cancer and slows down the time for developing from prostate cancer to androgen-independent prostate cancer and contributes to the improvement of quality of life.

## Figures and Tables

**Figure 1:** Analysis of patients' FACT-P quality of life scores and KPS scores ($\bar{\text{x}}$ ± *s*). Note: the horizontal axis indicates the scoring indicators, and the vertical axis indicates the value (points); after treatment, the FACT-P score and KPS score of the control group were (78.12 ± 7.85) and (62.18 ± 7.09), respectively; after treatment, the FACT-P score and KPS score of the experimental group were (91.03 ± 7.18) and (71.17 ± 7.23), respectively; ^*∗*^ indicates a significant difference in FACT-P scores between the two groups (*t* = 6.647, *P* < 0.001); ^*∗∗*^ indicates a significant difference in KPS scores between the two groups (*t* = 4.863, *P* < 0.001).

**Table 1:** Scoring standards of KPS.

Clinical symptom	Percentage method (points)
No evidence of disease	100
Minor signs or symptoms of disease; able to carry on normal activity	90
Some signs or symptoms of disease; normal activity with effort	80
Cares for self; unable to carry on normal activity or to do active work	70
Requires occasional assistance but is able to care for most personal needs; unable to do active work	60
Requires considerable assistance and frequent medical care	50
Disabled; requires special care and treatment	40
Severely disabled; hospital admission indicated	30
Very sick; completely disabled; hospital admission necessary; active supportive treatment necessary	20
Moribund; fatal processes progressing rapidly	10
Dead	0

**Table 2:** Analysis of patients' general information (*n* = 30).

Observation indicator	Control group	Experimental group	*X* ^2^/*t*	*P*
Age (years)	57.42 ± 6.38	58.04 ± 6.40	0.376	0.708
KPS score	64.02 ± 6.04	63.77 ± 6.12	0.159	0.874
FACT-P score	69.84 ± 6.65	70.15 ± 6.83	0.178	0.859
Duration of disease (months)	12.51 ± 2.56	12.84 ± 2.67	0.489	0.627
Number of chemotherapy (times)	8.05 ± 1.72	8.17 ± 1.69	0.273	0.786
Prostate volume (ml)	71.86 ± 3.28	71.93 ± 3.35	0.082	0.935
Gleason score	8.25 ± 1.17	8.34 ± 1.26	0.287	0.775
TNM stage				
II	11 (36.67)	9 (30)	0.300	0.584
III	18 (60)	19 (63.33)	0.071	0.791
IV	1 (3.33)	2 (6.67)	0.351	0.554
Pathological examination				
Good differentiation	7 (23.33)	8 (26.67)	0.089	0.766
Poor differentiation	16 (53.33)	17 (56.67)	0.067	0.795
No differentiation	7 (23.33)	5 (16.67)	0.417	0.519
CEA (*μ*g/L)	11 (36.67)	9 (30)	0.376	0.708
NSE (*μ*g/L)	18 (60)	19 (63.33)	0.159	0.874
CYFRA21-1 (*μ*g/L)	1 (3.33)	2 (6.67)	0.178	0.859

**Table 3:** Analysis of levels and ratios of TPSA and FPSA ($\bar{\text{x}}$ ± *s*).

Test indicator		Control group	Experimental group	*t*/*P*
TPSA (ng/ml)	Before treatment	80.47 ± 15.23	81.15 ± 15.81	0.191/0.849
	After treatment	55.71 ± 10.66	46.73 ± 10.28	3.321/0.002
FPSA (ng/ml)	Before treatment	8.26 ± 3.19	8.33 ± 3.53	0.091/0.928
	After treatment	5.14 ± 1.53	3.45 ± 1.28	4.640/<0.001
TPSA/FPSA	Before treatment	0.11 ± 0.06	0.12 ± 0.05	0.789/0.433
	After treatment	0.15 ± 0.06	0.20 ± 0.11	2.186/0.033

**Table 4:** Comparison of the situation of developing into androgen-independent prostate cancers of patients between the two groups.

Group	*n*	Number of affected patients	Time (months)
Control group	30	16 (53.33)	30.85 ± 7.24
Experimental group	30	8 (26.67)	39.71 ± 8.13
*X* ^2^/*t*		4.444	4.458
*P*		0.035	<0.001

**Table 5:** Analysis of patients' PSA level.

Group	*n*	<4 ng/ml	≥4 ng/ml
Control	30	17 (56.67)	13 (43.33)
Experimental	30	25 (83.33)	5 (16.67)
t		5.079	
*P*		0.024	

## Data Availability

Data supporting the findings of this study are available on reasonable request from the corresponding author.
